# Team-based Learning and the Analytical Skills of Medical Students as a Consequence of Increased Problem Difficulty

This article has been retracted.

**DOI:** 10.7759/cureus.4639

**Published:** 2019-05-10

**Authors:** Mustafa N Malik, Muhammad Abdullah Yousaf, Rida Riaz, Ahmed Ibrahim, Muhammad Abu Zar, Shehroz Aslam, Hafiz M Fazeel, Ceren Durer, Seren Durer

**Affiliations:** 1 Internal Medicine, The University of Arizona, Tucson, USA; 2 Internal Medicine, Rawalpindi Medical University, Islamabad, PAK; 3 Internal Medicine, Nawaz Sharif Medical College - University of Gujrat, Gujrat, PAK; 4 Internal Medicine, Rawalpindi Medical University, Rawalpindi, PAK; 5 Hematology and Oncology, The University of Arizona, Tucson, USA; 6 Internal Medicine, Maricopa Medical Center, Phoenix, USA; 7 Internal Medicine, Florida Hospital, Orlando, USA

**Keywords:** analytical skills, increased problem difficulty, problem solving, problem based learning, team based learning

## Abstract

Problem-based learning is a learner-centered teaching method, which uses real-world scenarios to promote student learning of concepts and principles. The aim of our study is to analyze the consequence of increased problem difficulty on team-based learning and the analytical skills of medical students. In our prospective descriptive study, two problem-based learning scenarios prepared on the topic of hypercortisolism were given to 197 students in two successive sessions. At the end of two sessions, the perceptions of students about team-based learning were documented using a five-point Likert scale on a standardized questionnaire for both scenarios (simple and complex) simultaneously. A written test consisting of multiple-choice questions (MCQs) and short essay questions (SEQs) was given at the end of a complex scenario to test the problem-solving skills and retention of knowledge. No statistically significant difference (p> 0.05) was noted in team-based learning between the simple and complex problem-based learning scenario. MCQs and SEQs of C-2 (interpretation) level were attempted well than C-1 (recall) level and C3 (problem-solving) level. In conclusion, the understanding of the problem by the medical students was improved; however, there was no significant improvement in the problem-solving skills and knowledge retention of the students.

## Introduction

Problem-based learning is a learner-centered teaching method that uses real-world scenarios to promote student learning of concepts and principles. In addition to knowledge acquisition, problem-based learning also facilitates the development of numerous other skills such as teamwork, problem-solving, information sharing, rational reasoning, mutual respect, and communication skills [1]. Problem-based learning scenarios are either simple or complex based on the difficulty level. Owing to the challenging nature of the problems, the development of skills to solve and, in turn, learn from them is crucial for human survival. The concept of problem-based learning was introduced by Howard Barrows at McMaster University in 1969, which was later adopted by various medical schools all over the world either partially or exclusively as part of their core curriculum [2].

Problem-based learning starts with formulating a problem in the form of a clinical scenario, which is usually integrated with both basic and clinical sciences [3]. An effective problem-based learning scenario should be naturalistic, in line with the pre-set learning objectives, engaging adequately with the intrinsic interests of the students, being able to excite the integration of knowledge across multiple disciplines, challenging, yet adjusted, to the student’s baseline knowledge, motivating to kindle the student’s discussion at a higher cognitive level, rational, open-ended, or designed in a gradual revelation model so that the discussion is not abridged too prematurely in the process, and planned in a milieu corresponding to student’s future career [4-5]. Complex problem-based learning scenarios are often challenging and provide students with an opportunity to look at the problem from various perspectives [6]. The amount of learning in a team is significantly greater than in an individual alone [7]. Problem-based learning provides a forum to work productively within a group setting and strengthen the team building skills of students [8]. The acquisition and retention of knowledge through problem-based learning can be determined using multiple choice questions (MCQs) and short essay questions (SEQs) test [9]. The aim of our study is to analyze the consequence of increased problem difficulty on team-based learning and the analytical skills of medical students.

## Materials and methods

In this prospective descriptive study, a total of 197 students were included. Two problem-based learning scenarios (simple and complex) were constructed on the topic of hypercortisolism. These scenarios were standardized through discussion by a group of teachers comprising subject specialists from both basic and clinical sciences in the context of the structure of the problem (simple or difficult), genuineness, relevance with the curriculum, brainstorming, and potential solutions. Students were divided into 14 groups, with each group consisting of 14 students. They were provided with these two problem-based learning scenarios successively, which were completed in two months. The easier scenario was given first and the difficult one was given afterward. At the end of a complex scenario, the perceptions of students about team-based learning were documented for both scenarios simultaneously using the five-point Likert scale (SD: Strongly disagree; D: Disagree; N: Cannot Comment; A: Agree; SA: Strongly agree) on a questionnaire comprising 15 items (Table 1).

**Table 1:** Assessment of team-based learning using a standardized questionnaire

N	Question Items
1	Motivation to participate in problem-based learning class was increased
2	Problem-based learning increased motivation to do well
3	Problem-based learning increased the comfort level for working in a team
4	Working in a team was better than working alone
5	When working alone, I did not learn as much as I did as when I worked in a team
6	Team-based learning takes less time
7	Team-based learning was not stressful
8	Team-based learning was a satisfactory way of learning the related content
9	Team-based learning taught me to work with students from different social, cultural and ethnic backgrounds.
10	Team-based learning is effective (i.e. learning happened)
11	Team Members freely shared information
12	Help from other team members benefited me
13	Teamwork made me more perceptive and sensitive to the needs of others
14	Team-based learning helped to make sense of areas that were still confusing after the lectures
15	Problem-based learning did not increase motivation to attend the problem-based learning class

At the end of the complex scenario, the retention of knowledge, interpretation of the problem, and problem-solving skills of students were tested by giving them a written test consisting of standardized nine multiple-choice questions (MCQs) and three short essay questions (SEQs). Standardized questions were prepared, which tested either of these attributes. The questions that tested knowledge retention were classified as “recall” level questions. The questions that tested the interpretation of the problem by students were classified as “interpretation” level questions and those testing the problem-solving skills of students were classified as “problem-solving” level questions. In this test, for every MCQ attempted correctly, a student would get one mark and for every SEQ attempted correctly, a student would get two marks. Paired Likert data about group learning items were analyzed using a Wilcoxon Signed Ranks test. A p-value of <0.05 was considered statistically significant. In the Wilcoxon Signed Ranks test, after tabulating the differences in the values of two samples, the values are ordered and assigned ranks from one through n to the smallest through the largest absolute values of differences. Then, a positive or negative sign is assigned to the ranks based on the signs of the observed differences. In our study, ‘a’ represents a positive difference, whereas ‘b’ represents a negative difference among matched pairs of question items one through 15.

## Results

The two problem-based learning assessments were compared using the Wilcoxon Signed Ranks test. No statistically significant difference was found between the simple and the complex problem-based learning scenario (p >0.05, z-score) (Table 2). At this point, the analysis is limited to only identifying the presence/absence of a statistically significant difference between the two testing items rather than the degree of difference.

**Table 2:** Comparison between complex and simple problem-based learning testing items using Wilcoxon Signed Ranks Test a: based on the positive ranks; b: based on the negative ranks.

	z-score	Asymp. Sig. (2-tailed)	Exact Sig. (2-tailed)	Exact Sig. (1-tailed)	Point Probability
Q1b - Q1a	-.769a	0.441	0.451	0.231	0.006
Q2b- Q2a	-.621a	0.545	0.539	0.261	0.005
Q3b - Q3a	-1.211a	0.231	0.229	0.123	0.003
Q4b – Q4a​​​​​​​	-.751a	0.461	0.461	0.218	0.005
Q5b - Q5a	-.299b	0.761	0.781	0.376	0.008
Q6b - Q6a	-.831b	0.438	0.421	0.205	0.006
Q7b - Q7a	-.921a	0.361	0.369	0.179	0.008
Q8b - Q8a	-.414a	0.681	0.681	0.31	0.005
Q9b - Q9a	-1.652b	0.110	0.111	0.051	0.001
Q10b - Q10a	-1.451b	0.157	0.150	0.069	0.001
Q11b - Q11a	-.491b	0.60	0.651	0.311	0.03
Q12b - Q12a	-.831b	0.411	0.411	0.210	0.002
Q13b - Q13a	-.621b	0.541	0.551	0.281	0.008
Q14b - Q14a	-.381a	0.711	0.721	0.348	0.008
Q15b - Q15a	-.191a	0.859	0.871	0.446	0.013

Effect size (ES) can be used to determine the degree of association between the groups using the ES formula in which |z| stands for the absolute value of z-score and N stands for the number of matched pairs included in our analysis. The ES ranges from zero to one. The cut-offs for the effect size to be considered small=0.10, medium=0.30, and large=0.50 were introduced by Cohen (1988), according to which the effect sizes that we calculated are very small (Table 3).

**Table 3:** Effect size between complex and simple problem-based learning testing items

	Effect size
Q1b - Q1a	0.04
Q2b - Q2a	0.03
Q3b - Q3a	0.09
Q4b - Q4a	0.04
Q5b - Q5a	0.03
Q6b - Q6a	0.06
Q7b - Q7a	0.07
Q8b - Q8a	0.04
Q9b - Q9a	0.10
Q10b - Q10a	0.08
Q11b - Q11a	0.04
Q12b - Q12a	0.07
Q13b - Q13a	0.03
Q14b - Q14a	0.04
Q15b - Q15a	0.02

Out of 197 students on the standardized multiple-choice questions (MCQs) written test, 128 (64.9%), 113 (57.3%), 141 (71.5%), 152 (77.1%), and 162 (82.2%) students attempted C2 (interpretation) level MCQ-1, MCQ-2, MCQ-5, MCQ-6, and MCQ-9 correctly, respectively, while 68 (34.5%), 83 (42.1%), 48 (24.3%), and 71 (36.1%) students attempted C1 (recall) level MCQ-3, MCQ-4, MCQ-7, and MCQ-6 correctly, respectively. Out of 197 students on the standardized short essay questions (SEQs) written test, 126 (64.04%) and 141 (71.53%) students attempted C2 (interpretation) level SEQ-1 and SEQ-2 correctly, respectively, while 73 (37.07%) attempted C3 (problem-solving) level SEQ-3 correctly (Table 4).

**Table 4:** Assessment of knowledge retention and problem-solving skills using standardized multiple-choice questions (MCQs) and short-essay questions (SEQs)

Total MCQs	Cognition Level of MCQs	Correct Answer
Not attempted		(2) 1.1%
1	C2 (interpretation) level	(128) 64.9%
2	C2 (interpretation) level	(113) 57.3%
3	C1(recall) level	(68) 34.5%
4	C1 (recall) level	(83) 42.1%
5	C2 (interpretation) level	(141) 71.5%
6	C2 (interpretation) level	(152) 77.1%
7	C1 (recall) level	(48) 24.3%
8	C1 (recall) level	(71) 36.1%
9	C2 (interpretation) level	(162) 82.2 %
Total SEQs	Cognition level of SEQs	Correct Answer
Not Attempted		16 (8.12%)
1	C2 (interpretation) level	126 (64.04%)
2	C2 (interpretation) level	141 (71.53%)
3	C3 (problem-solving) level	73 (37.07%)

## Discussion

There is little consideration of problem complexity among the issues in problem-based learning research. In general, subject specialist teachers or instructional designers use their experience-derived peerless verdict to establish an appropriate difficulty level for problem-based learning scenarios [6]. However, collaboration is paramount in the process of learning. After school life, there is a need for collaboration with others, sharing information and, hence, working more productively. The heart of problem-based learning lies in small group collaborations. ideally, a small group should not exceed 10 students [1]. However, due to logistic constraints, it was not possible for us to constitute groups of 10 students, and this can be one of the limitations of our study. Problem-based learning offers a unique forum for acquiring and nurturing the essential skills of team building and collaborative group learning in medical students. During a problem-based learning session, the instructor asks questions to make sure that the information pertinent to the group’s problem has been shared among the group members [1,8].

Studies focusing on the cognitive effects of problem-based learning show that the activation of previous knowledge, information recall, interpretation or theory formulation, and cognitive disagreements leading to conceptual change and mutual learning take place in the problem-based learning group. Studies focusing on the motivational effects of problem-based learning display that group discussion definitely impacts the students' built-in interest in the topic under discussion. The studies also reveal that a haphazard discussion in the problem-based learning group or a discussion that is superficial, perhaps caused by students being less motivated, restricts student learning in a small group [10]. Structuring problem-based learning problems with appropriate profoundness requires two parameters, complexity and ill-structuredness. If only basic information is required to solve a problem, the learners are expected to study the topic only frivolously. When a problem is easily resolved, the incentive and desire for the learners to probe deeper into the topic is slim [11].

Learning in the small group begins when students come across a real-life health problem that cannot be fully explained by them with the knowledge that they currently possess. Problems are plotted specifically to provoke interest and to create an eagerness to know upon, which students will act both individually and collectively. Problems may range in their level of difficulty, for example, following a user guide is a simple problem while assembling a car is a complex problem [12-13]. According to our results, no statistically significant difference (p>0.05) was observed between the perceptions of students regarding the effectiveness of group learning in a simple and a complex problem-based learning scenario but there is a need for more comprehensive research work to explore the effects of problem complexity on team-based learning activity. In Kitchener's model of cognitive processing, when individuals are faced with ill-structured problems, at the first level (level of cognition), individuals work out, memorize, read, recognize, and solve problems. At the second level (metacognitive level), individuals monitor their own advancement when they take on these first-level tasks. At the third level (epistemic cognition level), individuals reflect on the perimeter of knowing, the sureness of knowing, and the criteria of knowing. Assumptions based on the individual’s previous knowledge usually determine the individual’s ability to understand the problem and formulate an appropriate approach [14]. However, to obtain more information and to understand the cognitive and emotional effects of small group learning in problem-based learning settings, more research is required [10].

We can make group learning more fruitful by adopting the cooperative learning technique instead of simple discussion among group members. The cooperative learning method is an active educational approach with small groups for the purpose of both self-learning of the student as well as the entire group. A better understanding of the content learned is gained when students interact with each other and then clarify and discuss each other's insights on it. The effort to resolve potential disagreements during team collaborations leads to outcomes of quality reasoning, the precision of long-term retention and greater depth of knowledge, and a higher level of learning [15-16]. Cooperative learning is often used in the problem-based learning process. In one study, cooperative learning was administered in a problem-based learning course in a 10-week surgical clerkship and the difference of cooperative learning with conventional problem-based learning was evaluated. There was no statistically significant difference in outcomes between the study and control groups. However, in the cooperative learning group, students experienced that cooperation helped them learn, made studying more fun, and granted satisfaction, but they complained about the increased amount of time required by the group to work together, And it was not easy to perform group work with noise during the sessions [17-18].

A better score on the C-2 (interpretation) level compared to the C-1 (recall) level and the C-3 (problem-solving) level reflects that after going through difficult problem-based learning, students have shown better performance in C-2 (interpretation) level questions as compared to other level questions. However, there is a paucity of data to compare comprehensively our the results of our study with those of other studies. More prospective studies involving larger samples are needed to further explore the effect of problem complexity upon cognition level.

## Conclusions

No statistically significant effect of increasing problem difficulty was found in terms of team-based learning, analytical skills, and knowledge recall as is shown by the results of the C-3 (problem-solving) level and the C-1 (recall) level questions in the written test. However, difficult problems showed better results in terms of problem interpretation as is shown by the performance of students for the C-2 (interpretation) level questions. In conclusion, the understanding of the problem by the medical students improved; however, there was no significant improvement in the problem-solving skills and knowledge retention of the students.
